# Analysis of the Coordination Relationship between the Green Principle of Civil Law and Environmental Law in Environmental Pollution and Ecological Destruction

**DOI:** 10.1155/2022/2536704

**Published:** 2022-08-13

**Authors:** HuiJie Chai

**Affiliations:** Henan Police College, Zhengzhou 450046, China

## Abstract

Under the dual influence of environmental pollution and ecological damage, the green principles of civil law and environmental law can be better coordinated and developed. In the past, environmental pollution and ecological damage in the author's country were very serious. Hence, they designed and experimented with data extraction technology and environmental big data sets. A distribution model investigates it. Experiments show the following: (1) The system is developed from big data and can fully reflect the ecological environment of all parts of the country. Finally, it is concluded that the author's country's environmental pollution and ecological damage are very serious. (2) According to the experimental data of the figures and tables, it is concluded that the cooperation and coordination relationship between the green principles of civil law and environmental law not only has a protective effect on the ecological environment but also increases the economy of society and people. With the continuous updating and coordination of environmental laws and green prototypes, the author's country's environmental pollutants are significantly declining. The author believes that in the future, the country's ecological environment will become better, and the green principles of civil law will be more closely related to environmental law. The country's environmental pollution and people's lives are becoming more closely related. To better solve environmental problems, we have introduced the green principles of civil law and environmental law. It makes people's quality of life and the economy better. The main significance of the study is to use the method with the least damage to the environment to obtain the maximum economic benefit to achieve long-term sustainable development.

## 1. Introduction

This article illustrates that although antibiotics are therapeutic drugs for human beings, they are one of the important environmental pollutants. When antibiotics are applied to the human environment and agriculture, it is very likely that there are antibiotics that pollute the environment or antibiotic genes that produce antibodies in their residues. Their appearance has seriously affected the ecological environment of the microbiome in nature. The affected microorganisms are attached to the bodies of plants and animals, and they will soon pollute the natural environment and human environment [1]. This article describes the serious environmental pollution caused by industrial factors in Silesia, which leads to a very high probability of cancer and poor fertility in the region. Aromatic compounds on DNA and chromosomal mutations increase the risk of cancer and proliferation [2]. The article describes the prevalence of poor people who tend to live in areas with high levels of environmental pollution and environmental inequalities that affect human health and exacerbate epidemiological confounding factors. To investigate the impact of environmental pollution on people, we conducted research on different levels of environmental pollution in England. The results show that different pollutants bring different diseases to people, and the environmental pollution in rural and urban areas is very different [3]. This article describes the current situation and trend of environmental pollution in China. Although China is trying its best to control the air and water quality in cities, the environmental pollution problems in cities have not been improved much. China's sulfur emissions and nitrogen oxide emissions are rapidly increasing, however, CO2 emissions are taking the route of slowing down. Finally, the form of environmental pollution in China has always been very serious, and the future development of China will still depend on the road of industrialization [4]. This article introduces the problem of ecological damage caused by the combined water discharge and conducts water quality ecological surveys on rivers, such as the Odenwald and the Rhine Valley in southern Hesse, and it briefly discusses the follow-up of water quality ecology [5]. This article introduces that a lot of human and material resources are inseparable from the ocean area. People reclaim the sea at tidal and shallow sea locations to obtain more useful land area, however, this approach will seriously damage the coastal ecosystem, Therefore, an environmental economic model is constructed to analyze the damage caused by reclamation to the ecological environment, evaluate the value of marine space as a factor of production, and ensure the sustainable development of marine resources [6]. This article enumerates the damage to the original ecosystem caused by the introduction of foreign fish into the inland waters of Kenya. Although the introduction of new species will bring new economic benefits to the local area, it will not affect the carp in the waters and the lungs of Lake Baringo. The fish ecosystem is seriously damaged, and it is also a new challenge for the new economic trading system. How to balance the ecological damage and economic benefits has become the most important factor at present [7]. This article describes the serious pollution of the marine ecological environment caused by the oil spill in the Bohai Sea, which brings us a warning. To this end, the author's country has conducted a specific analysis of the existing laws and regulations on ecosystem damage, discussed the redefinition of marine ecological damage and the severity of penalties, put forward new suggestions, and improved the country's marine ecological damage laws [8]. To better investigate this article about biological invasions that can destroy local ecosystems and global biodiversity, the authors searched the Web of Science database to find information in the fields of entomology, agriculture, plant science, and ecology. The researchers have published articles covering biological control, risk assessment, weed control, pest control, and biological invasions and climate change in agricultural production. Based on these results, it is clear that more research is needed in Asia, especially in China. In addition, the impact of climate change on the characteristics of invasive species and the ecological destruction of invasive species ecosystems should be of greater interest in the future [9]. This article describes that to adapt to the green principles of the civil law, we use LID to reduce damage to the environment. Focusing on the balance between the environment and pollutants, LID will retain the water quality conditions of the development before design, and elements are retained in the design and planning. In addition to economic problems, LID also solves most of the environmental problems in the development process. The development system is currently the main promotion of the environmental protection law [10]. This article wants to fundamentally realize the green principle. For this reason, the green probability and principle of Anastas, Winterton, and Tang are cited to analyze the perfect solution, however, their green principle cannot clearly reflect the relationship between green and development, which also shows that these probabilities are not applicable, and there is still a long way to go in the optimization of economic benefits, effective mass yield, and green evaluation indicators around the green principle [11]. This article expounds the integration between green principles and humanization, analyzes the disadvantages of today's green products, integrates humanized design into the concept of green principles, enriches the content of environmental design, and expands the concept of environmental design. We strive to find the best combination of humanized thinking and green design, create a more complete framework for the green design strategy system itself, and implement the green concept into the entire product life cycle under the guidance of humanized thinking. Creative products promote the harmonious development of the environment [12]. This article mainly discusses the reasons why the author's country's environmental law has no effect on people. To see the current situation of the country's environmental law, the authors designed and established a system and historical background to give an overview of the environmental law, and finally, they came to the conclusion of China's environmental law. Deficiencies and concerns with respect to law enforcement tensions in the central and outer regions have been a major impediment to operations because of decentralization and increased regional protection [13]. This article describes the failure to achieve effective enforcement because of the continuous formulation and frequent revision of environmental laws in the country. The reason is due to the lack of legislative technology. Compared with many environmental laws and regulations, environmental standards are technical standards, and social reality has scientific and technological characteristics. Therefore, scientific progress can improve our understanding of environmental law causality. Technological advances can also update legal information and broaden the scope of legal solutions [14]. This article addresses the significant problem with environmental law that there is no information on the relevant public health and environmental impacts of industrial activities. Current laws do not counteract the conduct by not assessing the potential harm of their activities and by punishing them for doing so as a rule. It is the natural tendency of people to remain silent about the harm they can cause. Finally, some specific suggestions are given to reverse the impact of these unfavorable factors on the environmental law [15].

## 2. Environmental Law Analysis

### 2.1. Definition of Environmental Law

Environmental law is a general term for laws implemented in the country to protect the ecological environment and nature and reduce pollution and other harmful substances. The object of environmental protection is the land of the Chinese people, mainly soil, air, water quality, wetlands, grasslands, mineral resources, many natural environments, and so on. It includes man-made habitats, i.e., man-made environments, such as canals, reservoirs, plantations, historic sites, towns, and other settlements. The role of environmental law is to socially and economically divide the various social relationships involved in environmental protection and improvement created by people (including organizations) in production, livelihoods, and other reconciliation activities. It is to reconcile the relationship between social development and environmental protection. We must minimize pollution and environmental damage, balance the ecosystem, and complete the perfect integration of our people and the environment. There are two kinds of social relations in environmental law, one of which involves many relations related to the protection of natural resources, chemical pollutants, various wastes generated in life, and protection against harmful substances, such as garbage and noise. It is not difficult to understand that the environmental law is different from the emission control law, and titles, such as the emission control law, are limited to pollution prevention and management.

### 2.2. The Main Content of Environmental Law

The content of environmental law is very extensive, it includes the constitution and the comprehensive environmental protection law , which stipulates that protecting the environment and utilizing natural resources is the responsibility of all government departments, companies, and people. Achieve environmental goals together. According to the Greek constitution, the protection of the natural and cultural environment is the responsibility of the state. The constitution of the German Democratic Republic stipulates that the state and society, for the benefit of citizens, must do everything possible to protect nature, keep water and air clean, and keep the survival of animals and plants. It is also the duty of every person. Implement planned environmental management and incorporate environmental protection into social and economic development goals. The Soviet Union and Eastern Europe regard environmental protection as an integral part of their economic and social development plans, and maintaining environmental protection is also a top priority. Governments at the national and local levels should take necessary measures by taking it into account and seriously implement plans to avoid environmental pollution. Establish an environmental impact assessment system. The system requires authorities, companies, and institutions, as well as citizens, in the case of activities that have a significant impact on the quality of the environment to collect and study the natural and social conditions around them in advance and submit a written report. In principle, the polluter pays. The principle is that if the pollution affects it, the victim must be compensated and must bear the cost of cleaning up the consequences of the pollution. The pollutant discharge tax system and part of the pollutant discharge tax system are specific measures to implement the polluter-pays principle. The state provides financial information and tax incentives for environmental protection, environmental research, environmental scientific research, and other activities. In accordance with the requirements of the Japanese law, the government has adopted necessary fiscal and taxation policies, encouraged enterprises to build and improve pollution prevention facilities, and granted special benefits to small and medium-sized enterprises. Property tax exemption for environmental protection facilities tax exemption for land purchase, relocation to densely populated areas, etc. Illegal acts that threaten the environment shall be investigated for administrative, civil, and criminal responsibilities. There is a growing trend towards fulfilling this responsibility. For example, if damage is caused to human life, health, or property within the scope of damages caused by the discharge of substances harmful to the environment or health, the person responsible for the discharge will be liable for damages without negligence. In cases where criminal responsibility is pursued, the scope of responsibility has been expanded and penalties have been increased (in particular, increased penalties and longer sentences). According to the relevant laws of the Federal Republic of Germany, environmental crimes are punished on a 10-year basis. The burden of proof is in the plaintiff's favor and in the defendant's favor. The central government exercises an overall leadership in environmental work, and it has established special government environmental management agencies, such as the US Environmental Protection Agency, the Japanese Environmental Protection Agency, and the Environmental Protection Agency. Countries, such as the Soviet Union and Côte d'Ivoire, stipulate that environmental management must be carried out by corresponding institutions. All countries in the commercial sector emphasize and require local governments to be responsible for environmental protection work in their regions, and they will establish functional environmental management institutions. The content of environmental law is mainly to prevent environmental pollution and protect the environment and natural resources.

### 2.3. The Emergence and Development of Environmental Law

The environmental problems of human society a long time ago were because of the damage to the natural environment caused by agricultural activities. Later, with the vigorous development of the industrial market, industrial pollution started to occur. Some countries have taken partial measures since the mid-19^th^ century. The British Alkali Industry Act (1863), River Pollution Control Act (1876), Public Health (Food) Act (1907), River and Port Act (1910), and the French Air and Air Pollution Act No.48-400 have enacted corresponding laws to protect nature. For example, France, Austria, and Russia have developed a relatively complete forest protection legislation since the beginning of the 19^th^ century. The rapid development of the environmental law began in the 1950s and 1960s. The balance between natural resources and the destruction of ecosystems is getting worse. This would be a catastrophic pollution, and effective measures for environmental management include a formal set of environmental laws. It has grown into a new, independent legal institution.

### 2.4. Legal System

Today, in many industrially developed countries, the environmental law is already perfect, and it is an integral part of national law. The environmental law generally includes several aspects, such as legal provisions on environmental protection and environmental pollution. There are now environmental protection clauses in the constitutions of many countries. It is the highest standard and legal basis for state and social protection activities. There are regulations on the protection of land, minerals, grasslands, rivers, lakes, atmosphere, animals, plants, and natural environment, including regulations on the protection of nature reserves, historical sites, and national parks. Law and regulations for that prevention and control of air and wat pollution, noise and vibration, sedimentation, pollution, and other public hazards, including the prevention and control of odor and thermal pollution, the disposal of wastes, the management and control of pesticide, and other hazardous chemicals, and the prevention and control measures for radioactivity and electromagnetic radiation are provided. Different levels of environmental and hazardous conditions such as high water and high air levels involve legal protection issues. It emphasizes the establishment of legal liability, dispute and environmental system levels and various management methods, administrative law, criminal law, civil law, commercial law, labor law, and other environmental protection laws. In addition, some capitalist countries also include relevant judicial precedents.

### 2.5. Characteristics of Environmental Law

According to other jurisdictions, the environmental law, as an independent judicial body, has the following characteristics: environmental protection is the broad protection of the environment. The environmental law is not just an environmental law as it includes the constitution, environmental protection, criminal law, labor law, commercial law, and other laws. We must use scientific, engineering, and economic methods. The environmental law is closely related to the above methods. Therefore, the environmental law has many technical requirements. The environmental law is limited by economic and social systems. There are also laws targeting the natural ecology to protect natural environments, such as soil, air, water, and forests. As a legal branch, the environmental law expresses the will of the ruling class and contributes to its interests. However, it also adapts to different levels of social and national interests. The global environment in which human beings live is everything. Environmental problems are faced by all people, and we can learn from each other from the environmental laws of different countries.

## 3. Research on the Detection Method of Environmental Pollution and Ecological Damage

### 3.1. Environmental Pollution and Ecological Damage Emergency Risk Index Sampling

To accurately identify pollution and environmental hazards, the pollution control index is becoming a comprehensive technology for retrieving and disseminating information and protecting the environment. Big data and environmental risk index are used to establish an emergency pollution risk index model for environmental pollution and ecological damage. The correlation check and fuzzy clustering method are used to detect the emergency risk index of environmental pollution and ecological damage. Based on the risk index of data clustering model, the time-frequency distribution of emergency risk index of environmental pollution and ecological destruction is studied.

For the detection of environmental pollution and ecological damage emergency risk index, the correlation check, fuzzy clustering method, and filtering algorithm are used. The filtering algorithm can improve the environmental pollution detection ability and the emergency risk index. It fixes a linear kernel function to perform a set of rough set feature extraction, redundant filtering, and interference elimination on the extracted rough integrated features, and finally, the system also has the function of self-retrieval and error repair, which makes the research results of the system more reliable, thus realizing the algorithm and technology, which is of great help to the research on environmental pollution and ecological damage.

(1) $$\begin{array}{c} \begin{array}{c} p\left(t,f\right)=\int_{-\infty }^{\infty }s\left(u+\frac{\tau }{2}\right)s^{*}\left(u-\frac{\tau }{2}\right)\alpha \left(\tau ,v\right)\\ e^{-j2\pi \left(vt+f\tau -vu\right)}dudvd\tau , \end{array} \end{array}$$

(2) $$\begin{array}{c} \gamma \left(h\right)=\frac{1}{2}E{\left[Z\left(x\right)-Z\left(x+h\right)\right]}^{2}. \end{array}$$

The elements of risk index association rules are decomposed into time intervals, and the sample window is processed by feature selection and merging *n* ∈ [*n*_1_, *n*_2_]assuming that the two points are *n*_1_ and *n*_2_, respectively. The distance between the two points is designed to be normally distributed, and the statistical characteristics of the environmental pollution and ecological damage emergency risk index extracted from the existing framework can be calculated by the frequency estimation method to calculate the pollution response rate for statistical analysis. The formula for the sample value between the two points in the primary risk index is as follows:

(3) $$\begin{array}{c} \overset{\wedge }{w}\left(n\right)=\arg\underset{k\left(n\right)\in k}{\min}\left[\sum_{n=n_{1}}^{n_{2}}g\left(k\left(n\right)\right),k\left(n+1\right)+\sum_{n=n_{1}}^{n_{2}}fWVD\left(n,k\left(n\right)\right)\right], \end{array}$$

*p*(*k*(*n*); *n*_1_, *n*_2_). We have obtained the subsequent summary and treatment methods to successfully achieve the normalized adjustment of the emergency risk index of environmental pollution and ecological damage.

(4) $$\begin{array}{c} m_{i}\left(d_{l}\right)=\frac{\xi_{c_{i}}^{d_{l}}}{2\sum_{l=1}^{k}\xi_{c_{i}}^{d_{l}}-1}, \end{array}$$

(5) $$\begin{array}{c} m_{i}\left(\Theta \right)=\frac{\sum_{l=1}^{k}\xi_{c_{i}}^{d_{l}}-1}{2\sum_{l=1}^{k}\xi_{c_{i}}^{d_{l}}-1}. \end{array}$$

Formula (4) and formula (5) are the unified treatment of the emergency risk index of environmental pollution and ecological damage. Its purpose is to make the data better search, calculate, and reduce the time consumed by the system running. According to these formulas, the emergency risk index of environmental pollution and ecological destruction is analyzed, and the characteristics and correlation are explored according to the results of information sampling. Formula (4) represents the statistical summary of data in areas where the environment has been destroyed, and formula (5) is expressed as region division statistics for interference datasets. The proposal of these two formulas can make the collected environmental indicators more accurate.

where *l* = 1,2,…, *k*. The above formulas represent the sampling point *n*_1_ to the sampling point *n*_2_. The statistical value of the distribution of the emergency risk index between environmental pollution and ecological damage, defined as *k*(*n*)*g*(*x*, *y*) and*f*(x)the sum is in the formula*g*(*x*, *y*)for*k*(*n*). The cost function of environmental pollution and ecological damage, *g*(*x*, *y*) = *g*(|*x* − *y*|) relative to |*x* − *y*|, is characterized by a continuous time distribution. According to the above formula, the sampling of the environmental pollution and ecological damage emergency risk index is realized, and the characteristic profile and correlation exploration are carried out according to the information sampling results.

### 3.2. Finding the Characteristic Quantity of Emergency Risk Index

A distribution model of emergency risk indicators for environmental pollution and ecological destruction projects is established, a rough set of emergency risk indicators is extracted, and a correlation filtering algorithm is used to perform redundant filtering on the extracted rough set features. Disturbance elimination and pollution preparation for irrigation works. The frequency domain feature analytical structure model is used in the frequency domain space, and the method of minimizing the root mean square error estimation is used to check the risk indicators, and the function is tested through experiments. It shows that the method can improve the environmental pollution detection ability and improve the risk index of emergencies, and it fixes a linear kernel function to perform a set of rough sets of feature quantity extraction. The feature extraction rough sets of environmental pollution and ecological destruction emergency risk index satisfy the target set *POS*_*A*_^*∗*^(*X*) and the target feature negative field of the model *NEG*_*A*_^*∗*^(*X*). The data of the emergency hazard index satisfies the following:

(6) $$\begin{array}{c} POS_{A}^{*}\left(X\right)=\cup \left\{E|P\left(\frac{X}{E}\right)>P\left(X\right),\frac{E\in U}{A}\right\}, \end{array}$$

(7) $$\begin{array}{c} NEG_{A}^{*}\left(X\right)=\cup \left\{E|P\left(\frac{X}{E}\right)<P\left(X\right),\frac{E\in U}{A}\right\}, \end{array}$$

(8) $$\begin{array}{c} BND_{A}^{*}\left(X\right)=\cup \left\{E|P\left(\frac{X}{E}\right)=P\left(X\right),\frac{E\in U}{A}\right\}, \end{array}$$

In

(9) $$\begin{array}{c} P\left(\frac{X}{E}\right)=\frac{P\left(X\right)}{P\left(E\right)}=\frac{\text{card}\left(X\cap E\right)}{\text{card}\left(E\right)}, \end{array}$$

(10) $$\begin{array}{c} P\left(X\right)=\frac{\text{card}\left(X\right)}{\text{card}\left(U\right)}. \end{array}$$

card(*X*) represents the cardinality of the tracking set X under linear kernel operations. The continuous correlation filter detection method is used to establish the implicit function D (x) of the risk index distribution of emergency environmental pollution and ecological damage. At each sampling point, each X point in the pollution risk index distribution function has weighted information. In sample E, the rough sample points of the emergency risk index of environmental pollution and ecological damage s′, s′ is the nearest adjacent sample point of environmental pollution and ecological damage emergency risk index. If*s* ∈ *E*, theNearest(*E*, s′, *s*)。 is defined as follows:

(11) $$\begin{array}{c} \text{Nearest}\left(E,s^{\prime },s\right)\Leftrightarrow \forall s^{\prime \prime }\in E\left|s^{\prime }-s\right|\leq \left|s^{\prime }-s^{\prime \prime }\right|. \end{array}$$

At each sampling point, each s point in the pollution risk index distribution function has weighted information. Formula (11) indicates that there are two adjacent and nearest environmental pollution and ecological damage emergency risk index sample points in sample E that satisfy them, which belong to sample E. Then, there will be another point in sample E between the maximum range of the two points, and the definition formula of the Nearest of this point can be defined as formula (11).

The credibility of the environmental pollution and ecological damage emergency risk index supervision is as follows:

(12) $$\begin{array}{c} g\left(\frac{X}{E}\right)=\frac{P\left(X|E\right)}{P\left(X\right)}-1. \end{array}$$

The distributed information model of environmental pollution and ecological destruction emergency risk index *S* = (*U*, *C* ∪ *D*, *V*, *f*) is defined. Under the condition of association rules, the environmental pollution and ecological destruction emergency risk index is scored in score domain *NEG*_*C*_^*M*^(*d*)、boundary domain*BND*_*C*_^*M*^(*d*), and central domain*POS*_*C*_^*M*^(*d*). The formula is as follows:

(13) $$\begin{array}{c} POS_{C}^{M}\left(d\right)=\cup \left\{E_{i}|g\left(\frac{d}{E_{i}}\right)=\max\left(g\left(\frac{d_{1}}{E_{i}}\right),\ldots ,g\left(d_{m}|E_{i}\right)\right)>0,E_{i}\in E\right\}, \end{array}$$

(14) $$\begin{array}{c} NEG_{C}^{M}\left(d\right)=\cup \left\{E_{i}|g\left(d|E_{i}\right)=\min\left(g\left(d_{1}|E_{i}\right),\ldots ,g\left(d_{m}|E_{i}\right)\right)<0,E_{i}\in E\right\}, \end{array}$$

(15) $$\begin{array}{c} BND_{C}^{M}\left(d\right)=\cup \left\{\frac{E_{i}}{g\left(d/E_{i}\right)=0}E_{i}\in E\right\}. \end{array}$$

Formula (13), formula (14), and formula (15) are the environmental pollution and ecological damage emergency risk index check score domain, boundary domain, and central domain, respectively. After adding these three formulas, very bad and excellent ecological environment can be excluded. For environmental areas, it is the same as the principle of removing the highest and lowest scores when grading the competition. We set the ecological environment inspection score within a certain range to avoid the adverse effects caused by extreme data and ensure the ecological system calculated by the system. The environment is within the acceptable range, and it is not a common phenomenon in reality.

Finally, the Bayesian rough extraction results are obtained. In addition, adaptive planning and link extraction will be carried out according to the characterization results of the environmental pollution and ecological damage emergency risk index.

### 3.3. Detection Algorithm Optimization

On the basis of constructing the risk index distribution model of environmental pollution and ecological damage in emergencies, the risk index is collected, and a detection method for the risk index of emergencies pollution based on the original least square error estimation is proposed. The extracted coarse ensemble features are subjected to redundancy filtering and interference removal using a kernel-based correlation filtering algorithm. The gain function of the redundant filter is ∑_*l*=1_^*k*^max*g*_*ci*_(*d*_*l*_) ≥ 1 or∑_*l*=1_^*k*^max*g*_*ci*_(*d*_*l*_) ≤ 1. The statistical detection feature set of the kernel correlation filter satisfies the linear transformation of the instantaneous interference frequency with time, and the exponential detection adopts a function normalization method to detect, which is as follows:

(16) $$\begin{array}{c} m_{i}\left(d_{l}\right)=\max g_{ci}\left(d_{l}\right), \end{array}$$

(17) $$\begin{array}{c} m_{i}\left(\Theta \right)=1-\sum_{l=1}^{k}\max g_{ci}\left(d_{l}\right). \end{array}$$

where *l* = 1,2,…, *k*, for ∀*A*⊆Θ, Interfering with datasetsΘ, there are many mass function*m*_1_, *m*_2_,…, *m*_*n*_of rough set. The simple feature parameter extraction output is as follows:

(18) $$\begin{array}{c} \left(m_{1}⊕m_{2}⊕\cdots m_{n}\right)\left(A\right)=\frac{1}{1-K}\sum_{A_{1}\cap A_{2}\cdots \cap A_{n}=A}m_{1}\left(A_{1}\right)m_{2}\left(A_{2}\right)\cdots m_{n}\left(A_{n}\right). \end{array}$$

In,

(19) $$\begin{array}{c} K=\sum_{{}_{A_{1}\cap A_{2}\cdots \cap A_{n}=\emptyset }}m_{1}\left(A_{1}\right)m_{2}\left(A_{2}\right)\cdots m_{n}\left(A_{n}\right). \end{array}$$

Assume various characteristic attributes of x to be taken as *D*_*x*_=2. Then, we can get *ξ*_*c*_1__^*d*_2_^=3/5, *ξ*_*c*_2__^*d*_2_^=2/5, *ξ*_*c*_3__^*d*_2_^=2/5, maxg_*c*_1__(*d*_2_)=6/5, maxg_*c*_2__(*d*_2_)=3/8, and max*g*_*c*_2__(*d*_2_)=1/10. The frequency domain characteristic decomposition structure model for creating the emergency risk index of environmental pollution and ecological damage is as follows:

(20) $$\begin{array}{c} \min imize\left(\sum_{i\in v_{w},+}c_{0}^{w}\left|b_{i,0}^{w}+b_{i}^{w}\right|+\sum_{i\in v_{w,-}}c_{0}^{w}\left|b_{i,0}^{w}+b_{i}^{w}\right|\right), \end{array}$$

(21) $$\begin{array}{c} \sum_{e\in \delta_{w,-}\left(i\right)}x_{e}^{w}=\sum_{e\in \delta_{w,+}\left(i\right)}x_{e}^{w}+x_{i}^{w}\forall i\in \left(V_{w,+}+UV_{w,-}\right), \end{array}$$

(22) $$\begin{array}{c} \sum_{e\in \delta_{w,-}\left(i\right)}x_{e}^{w}=\sum_{e\in \delta_{w,+}\left(i\right)}x_{e}^{w}\forall i\in V_{w,=}, \end{array}$$

*C*_0_^*w*^ is the detection coefficient of the chirp, and *x*_*e*_^*w*^ represents the fluctuation of the pulse part. In the 2D plane (*m*, *n*), discrete sampling is used to obtain the cluster eigenvalues of the detection output of the environmental pollution and ecological damage emergency risk indicators.

(23) $$\begin{array}{c} \omega_{k}=\left(\begin{array}{c} v_{k}\\ e_{k} \end{array}\right)=\left(\begin{array}{c} x_{k}-f\left(x_{k-1}\right)\\ y_{k}-h\left(x_{k}\right) \end{array}\right). \end{array}$$

The above process realizes the algorithm and technology, which is of great help to the improvement of environmental pollution and ecological damage. However, when the algorithm is wrong, because the system data is too large and the calculation process is too long, the system will sometimes collapse. When we introduced a new formula, the system self-checks the wrong data.

(24) HX=px1Ix1+px2Ix2+n+pxnIxn=−∑i=1npxilogp2xi,

*p* represents the place where the error occurred in the system, *I* represents the time of self-discovery of the error, and finally, the statistics obtained the possible problems. Hence, the final result was obtained from the data, and then the result was placed in a special operation model. The correct data is calculated by the system as follows:

(25) $$\begin{array}{c} \frac{\partial E}{\partial W_{jk}^{\left(2\right)}}=\frac{\partial E}{\partial_{Y}}*\frac{\partial X}{\partial \Sigma }*\frac{\partial \left(\sum_{j}\partial W_{jk}^{\left(2\right)}*h_{j}\right)}{\partial W_{jk}^{\left(2\right)}}=2\left(\left|y-t\right|*P^{\left(2\right)}\left[\sum \right]*h_{j}\partial W_{jk}^{\left(2\right)}\right)=\partial W_{jk}^{\left(2\right)}-\alpha^{*}\frac{\partial E}{\partial W_{jk}^{\left(2\right)}}. \end{array}$$

Formula (24) will only have an impact when there is an error in the system. It can self-check the wrong place in the system and the time of self-discovery of the error, and then, it can put the obtained error result into the special operation formula (25) for correction. At this time, the manual help of the operator is needed, and the data before the error is obtained through simple data operation.

The overall process description of the environmental pollution and ecological damage emergency risk index is as follows: (1) the linear data is obtained from the transformation domain, and the average value is 0. (2) Define the narrowband interference identifier X⟶Z. (3) Set the number of components of the pollution emergency risk index to n. Recurrence k ← 1. (4) Randomly select the initial weight vector *W*_*k*_ to contaminate. Weighted adaptive learning to detect key risk cues. (5)*W*_*k*_ = *E*{*Zg*(*W*_*k*_^*T*^*Z*)} − *E*{*g*′(*W*_*k*_^*T*^*Z*)}*W*. (6) *W*_*k*_ = *W*_*k*_ − ∑_*j*=1_^*k*−1^(*W*_*k*_^*T*^*W*_*j*_)*W*_*j*_. (7) *W*_*k*_ = *W*_*k*_/‖*W*_*k*_‖. (8) Assume that*W*_*k*_does not satisfy the convergence condition, and step (5) is started. (9) Let *k* = *k* + 1k ≤ *n* and start step (4); (10) The system carries out self-correction of error data; (11) end..

## 4. Experiments and Conclusions of Ecological Environment and Environmental Law in the Green Principle of Civil Law

### 4.1. The Functional Orientation of the Prereorganization System under the Guidance of the “Green Principle”

Another “green principle” is to save resources, and the ultimate task is sustainable development. The “Green Principles” first appeared in the country's civil law system as Article 9 of the “General Principles of Civil Law.” The traditional concept of harmony between man and nature and elegant culture reflects the new concept of development put forward at the 18^th^ National Congress of the Communist Party of the country, and it reflects the country's densely populated national conditions. This demand has long resolved the contradiction between human ecology and resource ecology. From a judicial and economic point of view, resource protection must be understood in a broad sense. Not only as something generally accepted in court, but resource protection refers to the protection of a specific property or resource, and it is inclusive. This document adopts the interpretation of the “Green Principles” in the legal and economic sense. Prereorganization can enable enterprises to reduce the use of social and national resources, so that more economic resources can be invested in the ecological environment.

The primary goal of the bankruptcy law is to maximize the value of assets. We need to increase repayment rates for all creditors around the world and reduce the costs and liabilities of insolvency. We further recommend that to achieve this, a number of factors need to be considered. On the other hand, the value reduced by immediate liquidation of bankruptcy costs and the added value that bankruptcy reorganization can provide to creditors. Instead, assets must be preserved or improved. The amount of new investment and the cost of investment affect existing stakeholders. “Asset Maximization” aims to maximize returns on assets with low bankruptcy costs. It is a clear expression of legal and business “green principles”. “Prerestructuring” refers to reducing the restructuring costs and improving restructuring efficiency by considering the value of restructuring and the viability of debt businesses. The steps for a company to develop a plan before restructuring are as follows: if the company has financial difficulties, the company's management will negotiate with major creditors and major shareholders to resolve the company's current crisis. If the out-of-court negotiations are successful, the company's bankruptcy trend will be reversed. Debt acquires self-immunity, which is essentially a personal interest, however, the main disadvantage of personal interest is the “withholding” effect. A friendly negotiation can only be effective and carried out with the consent of both parties to the negotiation. If an individual creditor or multiple creditors choose not to encourage negotiation because the recovery rate has not improved significantly, or want to exercise their rights quickly, the settlement fails and lurks, and the victim disappears. Depending on the debtor's interests, prereorganization may provide legal enforcement to compel opposing creditors to comply with the agreement obtained. Therefore, the prerestructuring system is a perfect combination of public and private aid. It avoids the high cost and inefficiency of public funding, a disadvantage in terms of efficiency. The precalibrated system ignores the specifications of the fashion calibration system. The flexible and convenient negotiation process between topics reduces the negotiation time. Reduce negotiation costs, improve negotiation efficiency, and improve reorganization efficiency.  Figure 1 reflects the relationship between the number of prereorganizations of some enterprises and the ecoenvironmental economy.

There is an indirect link between the number of corporate prereorganizations and the ecological environment. The more the number of times of prereorganization, the higher the environmental and economic benefits. “Prereorganization” means that by considering the value of reorganization and the viability of the debt business, the cost of reorganization can be reduced and the efficiency of reorganization can be improved with the resource utilization of the country, so that more economic resources are put into the ecological environment. It is generally impossible to find their connection without a deep comparison between them.

### 4.2. Development of Environmental Law

Environmental law is very unstable, especially in the past 10 years. The revision rate of the country's environmental law has been very high. Environmental law is in disarray.  Table 1 shows some of the findings from the statistical period from 2011 to 2020. There are 10 laws amended or revised in the past 10 years, with a total of 18 revisions, with an average of 1.64 revisions per law. The natural resource conservation law was revised 3 times, an average of 4 times per law.

Logically, the destruction of current environmental laws is a combination of historical time and some social factors. It will not last long if the quality of the environment improves. However, eddy current damage is difficult to eliminate in a short time. These distractions do not just complicate law enforcement. It affects the law and safety, however, it also sends a “disturbing” message of environmental law. Inspired by “offensive” messages, interest groups seek to subvert media discourse. Guide public opinion, communicate relevant interests, and influence environmental legal procedures through repeated amendments to laws. Make the legal declaration that best suits one's interests. Achieving the goals of whether the environmental law is still “public” is unclear. Whether the “environmental law” can still protect the environment and avoid pollution has become a bigger problem.

Moreover, environmental law is still very complicated. Firstly, according to the legal statistics, environmental regulations account for about 10% of all laws, and environmental management regulations account for about 10% of all laws. It accounts for 7% of all prescriptions.Using the magic weapon of Peking University as the input database, there are currently 15 laws (including the Basic Law), 4 legal interpretations, 25 administrative regulations, 130 departmental regulations, and 1193 regulations in the country's current environmental protection laws. The Environmental Protection Act also includes local ordinances and Section 501 local government rules. Resource protection law rule consists of eight laws (except “protection of the marine environment”), one judicial interpretation, 20 administrative regulations, 594 local regulations, and 232 local government regulations. It is more intuitive than the previous data. Peking University's 110 legislation includes a lot of environmental protection laws. These figures reflect the environmental law. Secondly, adjusting for redundancy is important. Compliance with environmental laws is common.

Specific environmental factors are as follows: most of these environment entries go through several environment lists. Regulatory measures and governance goals are basically the same. It makes duplicate custom questions logical. For example, the groundwater natural resources and natural resources act regulates the extraction of natural resources. It includes groundwater extraction under the Water Resources Act. The two laws unwittingly overlap on regulatory issues. Of course, various environmental protection departments are also involved in comprehensive adaptation issues. Duplicate the custom question to see all the environments. Legal provisions vary. Some scholars believe that the repetition rate of various emission regulations in the environmental protection law exceeds 30%, especially in terms of performance. Pollutant discharge permits, emission standards, and equipment requirements comply with legal requirements. The author is from Peking University. Based on the legal comparison function of the miracle solution, it targets the relationship between specific environmental laws and creates the repetition probability of the graph array.  Table 2 clearly demonstrates this similar phenomenon.

The author's country's environmental laws do not exist independently. They are, more or less, related. Among them, the water pollution prevention and control law has the highest repetition rate with the other four environmental laws. Among them, the other four environmental laws have the lowest repetition rate. The concluded environmental laws include pollution sources of ocean, water, soil, atmosphere, and environmental noise, and the impact between them can also have an impact on others.

### 4.3. Analysis of the Ecological Environment of the Country's Previous Green Principle

As humans cut down a lot of trees, many forests have disappeared from the human environment. The lush Alps became a hopeless and desolate hill. Wild animals have lost their beautiful homes. Some species have become extinct, and the scene of people living in harmony with nature reminds us of the beautiful nature. If the forests are destroyed, then the world loses its natural layer of protection. Nutrient loss from soil increases in fertile areas, land degrades, and the ability of forests to withstand dust storms decreases. Forest air pollution diseases and infectious diseases are serious threats to human life. When the forest is destroyed, the sky is not blue, the mountains are not blue, and the water is not blue. The air is no longer fresh. There will be disasters, sandstorms, and a lack of water. The unbalanced ecological environment on which human beings depend has been severely damaged. It is urgent to rebuild the beautiful mountains and rivers and treat the damaged land. In view of these situations, Table 3 is the detailed analysis of environmental pollution we have collected, which can help us solve environmental problems more clearly.

Environmental pollution: although there are many kinds of environments, the way their pollutants are transferred to the environment are basically through the atmosphere, groundwater, plants, and soil. Therefore, if we want to solve environmental problems at this time, we can start from these four aspects. For the atmosphere, we can research and develop new products to purify air quality faster. Increase the control of groundwater discharge in the country, and set relevant laws and regulations to restrict people's behavior; in addition, plant more green plants that are beneficial to environmental protection.

Among them, the successful blockade of vegetation in dense forests can distribute rainfall. The rainfall intensity is greatly reduced, and the raindrops do not directly affect the land, absorb, nourish, and flow into the river, and they do not pollute the river. The water of the river is clear and blue, and the water quality is good. Because of the impact of human economic activities, the soil has lost its protection for wild plants. Much soil erosion makes the water turbid. A dry season and dilution because of deforestation can reduce the river flow. The purification capacity of the river is reduced, and the degree of water pollution is reduced. For the river environment, to make the water quality status easier for us to see clearly, we divided the water pollution levels into 6 grades (Table4).

There are various factors that cause environmental damage in our country. Among them, urban pollutant emissions are the most serious, followed by a large number of vehicle exhaust emissions. These pollutants are essential. We can only find ways to reduce these emissions or use other eco-friendly items to replace them. For now, the proportion of serious pollutants in the country is shown in Figures 2 and 3.

(1) For urban emissions: vigorously reduce citizen waste, reduce sewage discharge, utilize predischarge sewage treatment technology, develop and apply clean energy, reduce urban greenhouse gas emissions and the sound of car horns. (2) For vehicle exhaust emissions: make the country vigorously develop fuel substitutes, thereby reducing vehicle exhaust emissions, and vigorously develop clean energy vehicles, such as electric energy, solar energy, and wind energy. Optimize urban traffic road system: the optimized road can make cars take less detours and reduce emissions. Thus, the burning of energy in the car is reduced, and the smoother roads will continue to reduce the energy consumption of the vehicle.

At present, it can be concluded from Figure 3 that the country's environmental pollution problem can no longer be ignored. Problems, such as resource problems, land degradation, energy problems, and water shortages, are becoming more serious. People need to start on their own and improve their environmental awareness. Enterprises also need to enhance their sense of responsibility, strictly follow the national pollution and waste disposal requirements, and control the environmental pollution in the production process. The national regulatory agency needs to strengthen basic supervision and control. When pollution continues to increase, people will increase investment in scientific research to better solve the problem of environmental pollution in the country, and the environment can be continuously improved.

### 4.4. The Relationship between Environmental Law and the Green Principles of Civil Law

The environmental law manages social relations beyond the control of the civil code: firstly, the ultimate goal of the country's environmental law is to ensure sustainable social development. It is a form of law designed to be fulfilled, and it is difficult to incorporate the spirit of that law into the rights of all. Because of the economic conditions of the Chinese market at that time, it was difficult for civilians to engage in civil law activities. Therefore, the protection of certain individual rights related to certain environmental laws is a protection system suitable for the country's national conditions. The current social environment is likely to cause serious social problems and lead to the unfavorable implementation of the country's environmental protection policies. It requires the environmental law to fill the blank of civil law, mutual promotion, and joint promotion of ecological environmental protection. The green principle of civil law protects the personal and property rights of the victims of environmental pollution, controls the illegal acts of pollutants in accordance with the law, protects the ecological environment in principle, and reduces environmental pollution from the source. The civil law regulates social relations as a basic legal order to establish the correct codes of conduct according to the development of society, and the green principle applies to all citizens. It provides a legal basis for the subject of resource conservation and environmental protection, ensuring the successful realization of environmental benefits. The integration of environmental law and community law promotes the sustainable development of the environment: the essence of community law is every citizen's responsibility for environmental protection. Combining the legal environment with community rights requires both saving social resources and protecting and promoting the ecological environment. The sustainable development of society is the engine of development. Incorporate green principles into the civil code. The state is no longer the only institution protecting the ecological environment. Every citizen in society needs to be aware of environmental benefits. The above characteristics can be summarized through the renderings of their fusion in recent years. It is shown in Figure 4.

### 4.5. The Coordination Relationship between Environmental Law and the Green Principle of Civil Law and the Analysis of the Ecological Environment

Their mutual absorption and strengthening have led to a new improvement in the system. Environmental damage compensation system: compensation that can only be provided in accordance with the environmental damage tort law of the People's Republic of China is an incomplete remedy. However, the green principles go beyond these limits, and people feel their environmental rights are being violated. One can only get legal protection if one's personal or property rights are violated by environmental pollution. The country's civil procedure law does not define the status quo of environmental rights. However, the green principles define the environmental rights of citizens. For this, therefore, one can claim compensation for environmental damage if their privacy and property rights are violated. Ecological protection red line system: the ecological protection red line system creates a strict ecosystem protection system. Adhere to ecological security norms to ensure the coordinated and common development of ecological interests in the process of economic and social development. All civil law subjects have a protected environment. All citizens need to protect the ecological environment and monitor illegal activities that damage the environment. This strengthens environmental protection laws and expands the scope of the redline system. It has greatly helped the protection of the ecological environment: the country's investment in the environment has also greatly increased, and citizens' awareness of the environmental protection has been continuously improved. Various factors are developing in a positive direction. Figures 5 and 6 reflect the proportion of pollutants after the country's investment in recyclable waste and the integration of the two.

## 5. Conclusion

The theme of this paper is the analysis of the coordination relationship between the green principle of civil law and environmental law in environmental pollution and ecological destruction, which discusses the definition, main content, characteristics, and development of the environmental law. The author designed and experimented with the detection method of environmental pollution and ecological emergency risk index, calculated the characteristic quantity of serious environmental pollution, and concluded how to effectively solve the problem of environmental pollution. Although the country's environmental problems are serious now, the integration of the green principles of the civil law and environmental law will greatly reduce pollution problems. Not only the environment has been improved but also the laws and people's livelihood have been greatly improved. The author believes that in the future, the relationship between the country's green principles and the environmental law will become closer, and the environment will become more perfect.

## Figures and Tables

**Figure 1:** Prereformation and environmental economic links.

**Figure 2:** Proportion of pollutants discharged.

**Figure 3:** General proportion of pollutants.

**Figure 4:** The result of the fusion and coordination of the two.

**Figure 5:** Scale of recyclable waste in the country from 2013 to 2020.

**Figure 6:** The proportion of pollutants after improvement.

**Table 1:** Application of 4 laws in 2012–2020.

Legal name	2012	2013	2014	2015	2016	2017	2018	2019	2020
Air pollution prevention and control law	9	95	272	460	854	1516	2400	3194	2969
Water pollution prevention and control law	10	117	613	612	915	1655	1895	3464	2097
Circular economy promotion law	3	20	60	32	44	51	71	130	51
Cleaner production promotion law	3^*∗*^	3	6	3	7	4	4	6	4

**Table 2:** Partial duplication rate of provisions of environmental laws.

Legal name	Environmental protection law	Marine environmental protection law	Water pollution prevention and control law	Soil pollution prevention and control law	Air pollution prevention and control law
Environmental protection law	0	27.4	27.7	28.7	25.4
Marine environmental protection law	27.4	0	27.8	21.2	21.6
Water pollution prevention and control law	27.7	27.8	0	25.5	33.0
Soil pollution prevention and control law	28.7	21.2	25.5	0	26.2
Air pollution prevention and control law	25.4	21.6	33.0	26.2	0
Environmental noise pollution prevention and control law	25.0	19.0	17.0	15.2	18.5

**Table 3:** Environmental pollution analysis.

Environmental pollution incident	The way pollutants are transferred to the environment	Contaminant migration process	Receptor exposure pathway
Fire	Volatilize to atmosphere	Atmosphere-plants	Plant leaf respiration
Gas leak	Diffuse into the atmosphere	Atmosphere-plants	Plant leaf respiration
Discharge of pollutants	Discharge into groundwater	Groundwater-plants	Uptake by plant roots
Uptake by plant roots	Infiltrating soil	Soil-plant	Soil-groundwater-plants
Stationary waste accumulation	Particles and dust are dispersed into the atmosphere	Atmosphere-plants	Plant leaf respiration

**Table 4:** River pollution level table.

Pollution level	P1	P2	P3	P4	P5	P6
Water quality index	(0,0.2]	(021,0.4]	(041,0.7]	(071,1.00]	(1.01,2.00]	>2.00
Degree of pollution	It is good	Better	Light pollution	Moderately polluted	Heavy pollution	Heavily polluted

## Data Availability

The experimental data used to support the findings of this study are available from the author upon request.
